# Improving Patient Safety through Simulation Training in Anesthesiology: Where Are We?

**DOI:** 10.1155/2016/4237523

**Published:** 2016-02-01

**Authors:** Michael Green, Rayhan Tariq, Parmis Green

**Affiliations:** Department of Anesthesiology and Perioperative Medicine, Drexel University College of Medicine, Hahnemann University Hospital, Philadelphia, PA 19102, USA

## Abstract

There have been colossal technological advances in the use of simulation in anesthesiology in the past 2 decades. Over the years, the use of simulation has gone from low fidelity to high fidelity models that mimic human responses in a startlingly realistic manner, extremely life-like mannequin that breathes, generates E.K.G, and has pulses, heart sounds, and an airway that can be programmed for different degrees of obstruction. Simulation in anesthesiology is no longer a research fascination but an integral part of resident education and one of ACGME requirements for resident graduation. Simulation training has been objectively shown to increase the skill-set of anesthesiologists. Anesthesiology is leading the movement in patient safety. It is rational to assume a relationship between simulation training and patient safety. Nevertheless there has not been a demonstrable improvement in patient outcomes with simulation training. Larger prospective studies that evaluate the improvement in patient outcomes are needed to justify the integration of simulation training in resident education but ample number of studies in the past 5 years do show a definite benefit of using simulation in anesthesiology training. This paper gives a brief overview of the history and evolution of use of simulation in anesthesiology and highlights some of the more recent studies that have advanced simulation-based training.

## 1. Introduction

Anesthesia has often been compared to aviation industry [1]. Passengers entrust their lives to pilot, while patients undergoing anesthesia entrust their lives to the anesthesiologist. Both are high risk system with minimal tolerance for error [2]. Today the aviation industry has an exceptionally high safety record but this was not always the case. One of the most important reasons cited for the improvement in the safety of aviation industry has been the routine use of aviation simulators in the training of pilots [3]. Simulation is now considered a vital part of aviation industry culture to train pilots, air traffic controllers, and other flight crew. Simulation can similarly be used in anesthesiology curriculum to train residents.

Simulation in medical curriculum means recreating or imitating part of some clinical scenario for purpose of training or evaluation [4]. Simulation scenarios can be used for orientation to new procedures, exposure to uncommon clinical scenarios, and assessment of knowledge. Simulation accelerates skill acquisition, improves skill retention, and reduces the extinction of skills [5]. In addition to helping with the technical skills, simulation training can help reinforce nontechnical skills such as task management, leadership, team working, situation awareness, and decision making [6, 7]. These nontechnical skills are vital to patient safety in emergency and crisis situations. A usual simulation experience consists of three components: the initial briefing, the actual simulation experience, and the debriefing. Debriefing is the chief component of simulation that allows trainee to understand their decision making processes which is the first step in changing their clinical practice for better patient outcomes.

*Institute of Medicine* report on number of medical error [8] has focused public attention on better training, which has sharply increased the interest in simulation training. Today the cost of simulation has gone down significantly and it has become an integral part of anesthesiology residency training. The goal of this review is to give a brief overview of the history and evolution of use of simulation in anesthesiology and highlight some of the more recent studies that have advanced simulation-based training.

## 2. Methods

The study selection was performed using the MEDLINE, Scopus, and EMBASE database to find studies that investigated the use of simulation in anesthesiology. The search was restricted to English language (or English translation of) articles and abstracts published up to October 1, 2015. The search terms included the following: “Simulation”, “Medical simulation”, “Simulation training”, “M.E.T.I”, “High-Fidelity simulators”, “Anesthesia simulators”, “Patient simulation”, “Airway simulation”, “Anesthesiology simulation”, and “Anesthesiology residency simulation”. During the search, journal articles with topics related to testing of anesthetic equipment on simulation models were excluded. The results of the studies were divided by the different types of simulation training in anesthesia, that is, simulation of airway management, simulation of ultrasound guided regional anesthesia, use of simulation in obstetric anesthesia, and cardiothoracic anesthesia training.

## 3. Rationale for Using Simulation in Anesthesiology

Simulation is an interactive and innovative educational tool that can build confidence, improve clinical knowledge through practice, and enhance team performance. Anesthesiology is a hands-on specialty. As in other hands-on specialties such as surgery and emergency medicine, the only way to master a skill is to practice it again and again. Simulation provides a safe learning environment where anesthesiology residents and students can be taught, practice, and be evaluated on technical skills such as intubation and ventilation without ever putting a real patient at risk [9]. It is therefore not surprising that simulation has gained considerable interest and acceptance into anesthesiology education and curriculum. Anesthesiology is in fact the pioneer for the introduction of simulation into medical education [10]. Anesthesiology was instrumental in the development of a high fidelity human simulation used for medical education in other medical specialties as well.

The most widespread use of simulation in anesthesiology is to provide crisis management training. Simulation allows residents to experience clinical scenarios that are infrequent in daily practice, but critical to anesthesia practice such as the use of bronchial blockers and double-lumen endotracheal tubes (ETT) for single lung isolation. Failor et al. [11] enrolled 13 anesthesiology residents in a prospective, observational study to evaluate the effectiveness of using the high fidelity* AirSim Bronchi airway simulator* to teach residents how to manage lung isolation with double-lumen ETT and bronchial blockers. Instead of comparing resident performance before and after the simulation exercise, the authors noted the self-reported confidence of the residents with the devices. Resident confidence scores for each lung isolation technique improved after the simulation training, with the median gain ranging from 0.5 to 1.5. The largest improvement occurred with the bronchial blockers (*P* < 0.05), perhaps because, for many residents, it was their first chance to interact with a bronchial blocker. Simulation allows residents to get comfortable with rare anesthetic events. Simulation training improves skills and management when crises are subsequently presented in simulation environment. Bruppacher et al. [12] carried out a study to see if this translates into real life situations. The authors used weaning from cardiopulmonary bypass model to assess the effectiveness of simulation versus traditional teaching methods. Routine weaning from CPB is a high risk clinical setting involving a series of predictable technical and nontechnical clinical actions. The “simulation taught group” scored significantly higher than the “seminar taught group” at both 2 weeks (posttest) and 5 weeks (i.e., retention-test) on nontechnical skills global rating scale and a checklist of expected clinical actions, even though both groups performed similarly in the pretests.

Although the predominating use of simulation in anesthesiology is to educate in crisis management, it is also used to teach routine anesthetic management. Patient simulators can be used to recreate realistic environment and can help trainees practice routine skills for patient monitoring and the recognition and management of critical events, for example, while administrating sedation medications on patient simulators [13, 14]. In addition to anesthesiology residents, this simulation setup can be used to give hands-on training to nonanesthesiologists who routinely partake in sedation [15].

There are inherent limitations to teaching in the operating room; in addition to the natural distractions that hamper the learning experience, the balance between patient care and education needs to be considered. Resorting to simulation thus is the logical choice, which provides a platform for training in a risk-free environment. Simulation has been proven to be a helpful resource in training of not only anesthesiology residents but also the medical students rotating through the anesthesiology department [16]. Medical students can gain confidence by practicing airway and vascular access skills on mannequins before actually attempting them on a patient [17]. Similarly interactive group-based computer simulations in which students assume the role of anesthesiologist can improve their knowledge base of anesthesia [18].

After the ACGME mandated 80-hour workweek regulation for residents in US, educators are hard-pressed to find new and innovative ways to make the residency training experience as enriching as possible. Simulation is being used in new and novel ways. Aggarwal et al. [19] describe how they designed a* liver-transplantation anesthesiology simulation course* for residents at University of Pittsburg incorporating both traditional didactics and mannequin-based simulation. Outcomes of this intervention, as measured by pre- and postcourse quizzes, showed a statistically significant improvement. The residents also reported increased preparedness and confidence through self-reported questionnaires.

Simulation in anesthesiology has been used as an evaluating tool. There have been several studies assessing reliability and validity of simulation-based evaluation. Although in a few studies there has been some variability in reliability, especially on evaluating the behavioral aspects, on the whole there have been positive results regarding the reliability [20–22] and validity [23–25] of simulator-based evaluation when compared to traditional evaluation methods. It seems likely that in the future simulation-based evaluations could become a part of high-stakes examination. Devitt et al. [23] confirmed validity of simulator-based evaluations to differentiate a large group of individuals based on clinical experience or training. Over the coming years, the role of simulation as a training and evaluation tool in anesthesiology is expected to grow.

## 4. History and Evolution of Simulation in Anesthesiology

### 4.1. The Early Years

Although the use of simulation in medical education can be traced back to the medieval time, the first ever simulation model worth mentioning is “*Laerdal's Rescue Anne.*” It was a simple model designed to teach cardiopulmonary resuscitation. The first true moderate to high fidelity model in anesthesiology was made in the 1960s in University of Southern California. “*Sim One*” was a very expensive but life-like prototype with the anatomically shaped chest that moved with breathing, the eyes blinked, the pupils dilated and constricted, and the jaw opened and closed. The “Sim One” however had a very limited success as it was way ahead of it time and the technology at that time was not suitable to allow mass commercialization of this high fidelity model [26]. Around the same time, other mannequin simulators such as the “*Harvey cardiology mannequin*” were developed. This particular model could simulate up to 27 cardiac conditions [27].  Table 1 lists important milestone in history of simulation in anesthesiology.

### 4.2. Introduction of Software Based Simulation

As the mathematical models of physiology and pharmacology became clearer, various computer software attempted to simulate the normal human response.

In 1982 Philp JH introduced the* Gasman* software for teaching the pharmacokinetics of anesthesia administration. It calculates the time course of anesthesia uptake in each compartment of the body as well as the breathing circuit and vaporizer. Since its introduction more than 33 years ago, an updated version of Gasman (Med Man Simulations, Inc., Boston, MA) is still in use in residency training programs across the country [28]. Daniel et al. [29] demonstrated how the use of this pharmacokinetics software, Gasman, objectively improved the understanding of pharmacokinetics principles in 23 residents.

*Anesthesia Simulator Consultant* [30, 31] was developed by* Schwid* in the late 1980s to simulate critical events in anesthesia and critical care. It is still being used with minor updates in its software.

### 4.3. High Fidelity Mannequin Simulators

In 1987, Dr. David Gaba at* Stanford University* developed a very realistic, physical simulation system which he labelled* CASE 1.2* (Comprehensive Anesthesia Simulation Environment). CASE was built primarily to help with Anesthesia Crisis Resource Management (ACRM) training [32].

Around the same time, Dr. J. S. Gravenstein and his colleagues at University of Florida created the* Gainesville Anesthesia Simulator (GAS)*. It was a very sophisticated simulator that could imitate breathing and generate a pulse, EKG, and a lung that followed normal physiological calculations to consume and eliminate gases accurately. There were hidden sensors on the functionally intact anesthesia machine that recorded users' action which were used in providing feedback [33, 34].

Around the 1990s, a number of commercial high fidelity anesthesiology simulators (HFS) were introduced based on the principles of the above two HFS. The simulators in use around the world today are updated versions of the same simulators.

## 5. Current State of Simulation in Anesthesiology

At the present time, there are about 80 commercially available simulators for use in anesthesia, with prices ranging from 100 US $ for the software based simulators to more than 50,000 US $ for the high fidelity patient simulators. Cumin and Merry [35] classified these commercially available simulators based on the following 3 categories:

1. Mode of interaction (screen-based, hardware-based, or virtual reality-based).
2. Physiological model used.
3. Their use to teach predominantly psychomotor skills or cognitive skills.

Of special interest are the following high fidelity patient simulators that are in wide use in anesthesiology residency training programs around the world.

*SimMan™* (Laerdal, Stavanger, Norway) is an advanced patient simulator that has a realistic airway, allows vascular access with pharmacological drug recognition system, and can even display neurological or physiological symptoms such as seizures and tears. Teatherless operation allows the educators to monitor the performance of the trainees remotely through a variety of clinical scenarios. SimMan is capable of simulating normal and difficult airways and also testing of airway equipment.

*HAL*®* Patient Simulator* (Gaumard, Miami, Florida, USA) is another similar high fidelity simulator in use today [36]. It boasts programmable airway, realistic vital signs, and blood pressure and allows performance of tracheostomy or needle cricothyrotomy [37].

*METI-Human Patient Simulator* (CAE Healthcare®, Sarasota, Florida) has a very detailed cardiovascular, respiratory, neurological, and pharmacological modeling and claims to accurately represent complex critical care and drug interaction scenarios [36]. Different add-ons of Human Patient Simulator (HPS) allow for simulation of central venous cannulation [38] and arterial cannulation.

Several studies have tried to determine the accuracy of these high fidelity simulators. Lejus et al. [39] evaluated the accuracy of the METI-Human Patient Simulator during oxygen administration and apnea maneuvers. They found that* O2 pulse saturation (Spo2) on HPS decreased much later when compared to human subjects, regardless of preoxygenation*. Schebesta et al. [40] evaluated the upper airway anatomy of four high fidelity patient simulators and two airway trainers in comparison with actual patients (*n* = 20) by means of CT scan. The METI-HPS (METI®, Sarasota, FL) was found to be the most realistic high fidelity patient simulator with regard to accuracy of airway parameters (6/19 [32%] of all parameters were within the 95% CI of human airway measurements). Hesselfeldt et al. [41] concluded that SimMan patient simulator was “*acceptably realistic*” for simulating mask ventilation, laryngeal mask insertion (LMA), and endotracheal intubation. They did however point out some of the shortcomings of SimMan such as* difficulty in maintaining a mask seal and the shortened distance from teeth to the vallecula*.

A recent randomized control trial [42] compared the currently used high fidelity simulators, SimMan, and HAL Patient Simulator to actual patients. The performance of endotracheal intubation was found to be comparable in patients and both simulators. However for LMA, no chest rise was visible in 35% (HAL) and 32.5% (SimMan) of the cases after inserting LMA. Furthermore, effective mask ventilation was not possible in 60% of the cases using HAL, compared with 0% of cases using SimMan and 2.5% of patients (*P* < 0.001). This study questions the validity of currently used simulators for supraglottic airway management techniques but does suggest that they have good validity for endotracheal intubation.

Future models of high fidelity simulators could address this issue in construction and allow for more realism in supraglottic airway management techniques. The fact remains that no patient simulator, no matter how technologically advanced, can ever mimic the human body perfectly. It is important however to recognize these limitations and the differences and limitations of the simulators should be given due consideration during the debriefing process.

## 6. Finding the Balance between High versus Low Fidelity

The fidelity of a simulator is the degree to which the simulator replicates the real environment [43]. High fidelity mannequin simulator imitates human physiology and anatomy as realistically as possible, compared to a low fidelity CPR model. It is often assumed that the high fidelity simulator gives a richer training experience. However, this might not always be true. This also depends on a large part of the objective the educators are trying to achieve. This was shown by Nyssen and colleagues when they compared effectiveness of computer screen-based simulators and effectiveness of mannequin-based simulators [44].

Chandra and colleagues studied the effectiveness of a low fidelity versus high fidelity fiber optic intubation training model. There was no significant difference between the low fidelity (*n* = 14) and high fidelity (*n* = 14) model groups when comparing the global rating scale, checklist, time, and success at achieving tracheal intubation [45]. Similarly Friedman et al. did not find any advantage of using HFS on pediatric residents' airway management and intubation skills when compared to low fidelity model. Other studies [46] evaluated the effect of training on high fidelity versus training on low fidelity epidural simulators on the residents' performance. Two blinded observers graded the videotaped performance of residents performing epidural anesthesia on patients. No significant difference could be found between the group that was trained on high fidelity simulator and the group that was trained on low fidelity simulator. A recent meta-analysis of 14 studies looking at the benefit of using high fidelity model for advanced life support training showed no significant improvement over low fidelity models with regard to either the skills or the knowledge [47].

Although most of these studies evaluating low fidelity versus high fidelity simulation training are small, low-powered studies and their results should be interpreted as such; however, it seems that under certain circumstances the benefits of simulations can be reaped by using a more economical approach. Even anesthesiology residency program with financial constraints can employ low-cost, low to moderate fidelity solutions and still achieve comparable results. Anesthesia departments across the world are trying to experiment with low-cost, high fidelity model. Hartwell et al. [48] described how they fashioned such a machine in New Zealand using biomedical calibration machines and modified basic manikins already available in the institution.

In the future, the more expensive, high fidelity simulators should be compared with the more economical low fidelity simulators and a cost to benefits ratio should be calculated to see if they provide any real advantage over the already available simulation devices. The key is to use the appropriate fidelity model based on the expected educational and learning objectives [49].

## 7. Simulation in Airway Management

Difficult airway management is one of the primary challenges and most important patient safety issue in the practice of anesthesiology. It is the leading cause of death and legal ramifications in anesthesiology [50, 51]. It is vital that anesthesiology residents receive the best possible training in airway management. Airway management is primarily a psychomotor skill; hence simulation training seems a very suitable way to teach such skills [52].

ASA has published algorithms on management of difficult airway [53]. In case of a “can't intubate, can't ventilate” (CICV) scenario, transtracheal oxygenation and cricothyrotomy are the final options. But these are rarely practiced by physicians in real life, yet every anesthesiologist should be extremely proficient in these lifesaving technique. Simulation training is ideal way to teach anesthesia residents the hand-on skill of cricothyrotomy. This can be done either on high fidelity simulator with the replaceable/consumable trachea and skin or on cow cadavers. Hubert et al. [54] evaluated the effects of high fidelity cricothyrotomy simulation on compliance with difficult airway management algorithms and the technical skills of cricothyrotomy.* 27* anesthesiology residents were recruited to the study. The participants took a “preintervention simulation test” based on CICV scenario simulator in which only 63% of the residents adhered to airway management guidelines. The residents were taught the principles of difficult airway management in a 2-day seminar including hands-on training on a task trainer. Postintervention tests which were done randomly at 3, 6, or 12 months after the simulation training session showed that 100% of the residents adhered to the guidelines and there was improvement of duration and technical quality of the cricothyrotomy. A similar earlier study by Boet et al. [55] showed similar results and a retention of skills when tested a year later. It is interesting to note the retention of complex psychomotor skills acquired through simulation.

Fiberoptic orotracheal intubation (FOI) is a complex psychomotor skill indispensable to the practice of anesthesiology. However residents often have a limited experience to practice FOI on real patients. Simulation can cover this gap in training. It is known that FOI intubation skill can be learnt outside the OR [56]. Several studies have evaluated the FOI simulation training.

Nilsson et al. [57] studied 23 anesthesia residents in a randomized controlled study to evaluate simulation-based training in FOI. They tried to determine the optimal structure of training, that is, dividing the training either into segments (part-task training) or at once (whole-task training). Residents were allocated randomly to receive either part-task or whole-task training of FOI on virtual reality simulators. Procedures were subsequently evaluated on a mannequin. They were then compared to experienced anesthesiologists who had no prior such training. They found that a positive learning effect was observed in both the part-task training group and the whole-task training group and that part-task versus whole-task training did not seem to make a difference (*P*  =  0.61).

In a recent meta-analysis of advanced airway management simulation training, Kennedy et al. [58] evaluated 76 observational studies and trials (total: 5,226 participants). Simulation training was compared with both no intervention and nonsimulation intervention. Simulation studies compared with no intervention showed a benefit of simulation in improving knowledge and skills,* but not in behavioral or patient outcomes*. Simulation compared with nonsimulation interventions showed increased learner satisfaction and improved skills and patient outcomes (in a very limited number of studies, *n* = 3) but not knowledge. However this meta-analysis was subject to heterogeneity and variation among included studies.

## 8. Simulation in Regional Anesthesia

Over the past few decades, regional anesthesia has become synonymous with the use of ultrasonography (US) [59]. Simulation is an effective tool, proven to help anesthesiology residents get comfortable with the use of US in regional anesthesia techniques. A study was carried out at University of California at Irvine Medical Center (2014) to test the effectiveness of US compared to traditional didactic lecture. In this prospective, blinded trial, 20 anesthesiology residents were allocated to either traditional 90-minute one-on-one didactic lecture or a 90-minute training in a simulation center to learn the same topic. No differences were noted between the two groups in prelecture test scores (*P* = 0.97). The simulation group however showed higher scores on both the postlecture multiple choice (*P* = 0.038) and postlecture human-model examinations (*P* = 0.041) as well as a greater overall interest in perioperative ultrasound (*P* = 0.047) [60].

Woodworth and his colleagues designed a similar, single center, prospective study in which 29 participants were randomized to either* simulation group* in which teaching video with interactive software simulation was used or* control group* in which sham video was used. Participants were tested before and after simulation training, on their ability to identify anatomic structures on US images, as well as their ability to locate the sciatic nerve with US on live models. A 25-minute instructional video and a software based interactive simulation considerably improved knowledge of US anatomy of the sciatic nerve; however there was no significant improvement in the live US scanning skills [61]. While the study had several limitations including lack of a validated assessment tool for US image interpretation skills and small sample size, it is interesting to note that the improvement in knowledge did not directly translate into improved skills in ultrasonography. Niazi et al. [62] observed that an hour long simulation training on needling and proper hand-eye coordination improved subsequent clinical block success. Several other studies have demonstrated an objective improvement in US skills in UGRA after simulation training [63–65].

Simulation has been proven as a helpful tool not only in teaching adult USRA but also for teaching pediatric USRA. A novel curriculum with integrated simulation model for teaching and evaluating UGRA skills in pediatric anesthesia fellows showed promising results. Over the course of academic year, cognitive UGRA-related skills of trainees improved from baseline results of 53% to 79% at 12 months [66]. All this recent literature shows a benefit of integrating simulation training for improving the knowledge base and to a limited extent the psychomotor skills involved in UGRA. The American Society of Regional Anesthesia and Pain Medicine (ASRA) and European Society of Regional Anesthesia and Pain Therapy (ESRA) have published joint committee guidelines for training in UGRA. These guidelines encourage the use of simulators and phantom models in UGRA training [67]. However more research is certainly needed to optimize the use of simulation in regional anesthesia training [68].

## 9. Simulation in Obstetric Anesthesia

Obstetric floor can be a challenging environment for many anesthesiology residents. The anesthesiology residents have to hone their skills in a short duration of time, in a high risk setting. Thus like other anesthesiology subspecialties, simulation provides the perfect training ground. There are four broad uses of simulation in obstetric anesthesia: improvement of technical skills, nontechnical or teamwork skills, individual clinical competence, and the safety of the clinical environment [69, 70]. Technical skills such as epidural anesthesia and estimating volume of blood loss [71, 72] can be effectively taught via the use of simulation. Similarly videotaped simulation sessions can be used to teach team communication skills [73].

The volume of cesarean deliveries done under general anesthesia (GA) has significantly diminished over the past few decades. Educators have advocated to use simulation training to fill this gap in training of the residents [74].

Scavone et al. [75] described a standardized scoring system for objective assessment of residents' performance of GA for emergency cesarean delivery on high fidelity simulator (HPS). This tool was found to be both reliable and valid. Using this scoring system Ortner et al. [76] compared 24 residents to obstetric anesthesia attending physicians. The residents were exposed to repeated simulation-based training programs to perform GA for emergent cesarean delivery, over the course of 8-week obstetric anesthesia rotation. The residents showed a measurable improvement in performance. It was also interesting to note that the objectively measured performance scores remained almost at the same level 8 months later showing long term retention of simulation acquired skills.

Similarly, another study by Scavone at al. testing the effectiveness of focused simulation-based training on emergency obstetric anesthesia showed encouraging results. Residents exposed to the simulation group showed higher objective scores in the preoperative assessment, equipment availability check, and intraoperative management and higher score overall as compared to the control group [77]. This study shows a clear advantage of obstetric anesthesia simulation training on clinical performance but further studies in the field should explore the advantage of simulation training on residents' performance on actual patient.

In addition to helping with technical skills training, simulation is the ideal environment to teach essential skills needed to function as a team such as communication behaviors, leadership skills, collaboration, and role clarity [70]. Obstetric crisis is the ideal platform for team training exercises because of the acuity of the medical conditions, the interplay of different medical personal involved, and the importance of timely communication [78]. Several authors have studied the role of simulation in refining team work skills [79, 80]. They found that simulated obstetric emergency was perceived positively by the participants and it caused a measureable performance improvement in the simulated environment; however it is not known if that translates into actual clinical performance.

There has been a lot of recent interest in the use of simulation in obstetric anesthesiology as evident by literature. In addition to some of the above studies, there have been several reviews [69, 70, 81] on the topic as well as instructional articles [82, 83] that guide how to best perform specific simulation in obstetric anesthesiology. Recently specific “task trainers” for spinal anesthesia [84] and epidural anesthesia [85] have been described, albeit not perfect. Future models of these specific task trainers can build upon the experience gained and make improvements in the construction that can improve the validity of the training as compared to actual human anatomy and physiology.

## 10. Simulation in Cardiothoracic Anesthesia

With the recent technological and research advances, cardiothoracic and vascular anesthesia is becoming increasingly complex. Trainees have to learn intricate skills in a short period of time. Simulation allows them repeatedly to practice such skills and management of complex cases in a low-stress environment without putting actual patients in harm's way. Simulation is certainly a valuable addendum to the routine training in cardiothoracic anesthesia [86].

In addition to the high fidelity patient simulators mentioned above, there are several simulation devices available in cardiothoracic (CT) anesthesia. These function either as stand-alone devices or as an add-on to HFS. These include devices to practice skills such as central venous line cannulation such as* Lifeform Central Venous Cannulation Simulator (Nasco, Ft. Atkinson, WI)* and the* Louisville Central Venous Cannulation Simulator* [38]. Similarly there are devices to simulate arterial cannulation which are constructed from molded plastic or latex with a rubber tubing placed within the artificial limb and also have a mechanism for generating “arterial pulsation” (either with a manually squeezed or electronic pump) [87]. While these devices can only approximate normal anatomy, but nonetheless they are useful for teaching the actual procedural steps in cannulation, the interpretation of the data derived from the monitor, and any simulated complications. Another interesting device, although not commercially available, is* Sydney Perfusion Simulator (Ulco Engineering, Marrickville, Australia).* It is a software-controlled, electrically driven hydraulic device. It was developed to reduce the incidence of serious errors in the use of cardiopulmonary bypass [88].

Bronchoscopy is a useful skill for anesthesiologists when dealing with complex cases involving difficult airway and lung isolation and when working in critical care unit. It is therefore necessary that an anesthesiologist should be adequately skilled at bronchoscopy. In addition to the cognitive ability, excellent manual dexterity and hand-eye coordination are needed to get meaningful results from a bronchoscopy [89]. Simulation training is the ideal means to practice these skills. Bronchoscopy simulators vary in design from simple nonanatomical box trainers [90, 91] to virtual reality-based bronchoscopy simulators [92]. Several studies have shown the benefits of using a simulation-based bronchoscopy curriculum [93–95]. The choice of the bronchoscopy trainer used depends upon the desired learning objectives.

In the ever-changing landscape of anesthesiology, where the anesthesiologists are assuming the role of perioperative physicians, the utilization of transesophageal echocardiography (TEE) and transthoracic echocardiography (TTE) is increasing. Simulation is a helpful way to teach basic concept of TEE. It has been shown to improve cognitive skills like normal echocardiographic anatomy, structure identification, and image acquisition [96, 97]. In a recent study Ferrero et al. [98] showed how mannequin-based TEE simulation training allowed residents to obtain significantly higher-quality images, compared to control group who received conventional didactic training in TEE. Over the past few years, several studies have evaluated the validity of echocardiographic simulation devices with overwhelmingly positive results. In a similar randomized study design, Neelankavil et al. [99] showed how anesthesiology residents showed better cognitive appreciation of transthoracic echocardiography (TTE) when trained on TTE Simulator* (Heartworks, Inventive Medical Ltd.)*, compared to control.

All these studies do show an advantage in using simulation in CT anesthesia, although more research is certainly needed to explore this topic further. It seems likely that simulation training will continue to integrate itself in cardiothoracic anesthesiology training alongside the conventional didactics.

## 11. Teaching Nontechnical Skills Using Simulation in Anesthesiology

Recently there has been a lot of interest in using simulation to teach and evaluate nontechnical skills. Nontechnical skills encompass skills such as communication skills, interpersonal skills, and team management [100]. While these skills are not necessarily acquired through routine clinical training, yet these are important for an anesthesiology resident to learn these skills. Nontechnical skills can be improved by the use of patient actors and videotaped encounters can be used to evaluate, analyze, and give feedback of any communications training or intervention [73, 101]. However, compared to other medical specialties, anesthesiology relies less on the use of “standardized patients” due to the intrinsic nature of the anesthesiology and difficulty in arranging and training the so-called patient actors [102].

Howard and colleagues described the anesthesia crisis management training which they called “Anesthesia Crisis Resource Management” (ACRM) based on Crew Resource Management (CRM) used in the aviation industry for crisis situation [32]. The participants were given didactic instructions on the relevant topic before the simulation experience in the actual OR. This simulation was videotaped and used in the debriefing session. The idea is to put the resident in an actual OR setting and the actions are observed from another room, as not to become part of the scenario. There was an objective improvement in knowledge about anesthesia crisis management after the first course (but not the second course). This was the first time nontechnical aspects of anesthesiology were thoroughly analyzed in regard to a simulated situation. The principles of ARCM have been taken up by other centers around the country and internationally in countries such as Canada [103], UK [104], Germany [105], and New Zealand [106].

Since then several studies have described how the use of patient mannequins and HFS can build essential nontechnical skills such as team work. Yee et al. [6] have described how only a single session of training on high fidelity mannequin simulator improved the nontechnical skills of anesthesia residents as measured by the standardized* Anesthetists' Nontechnical Skills (ANTS) system*. Paige et al. [107] conducted a small scale pilot study to understand the effects of high fidelity simulation-based,* interdisciplinary* operating room training on team communication skills and crisis-related teamwork. Majority of participants self-reported it as a useful experience that will change their clinical practice. In another study, the results objectively showed an improvement of* self-efficacy for effective teamwork performance in everyday practice* [108]. However these studies depended on self-reporting, which is subject to inherent bias and therefore should be interpreted with reasonable degree of caution.

## 12. Translation of Simulation Training into Patient Outcomes

The current level of evidence supports the use of simulation techniques in the training of anesthesiologists. Simulation training is known to increase not only self-reported confidence [107, 108] but clinical performance as well [109]. It is reasonable to hypothesize that the results of improved clinical performance would reflect as improved patient outcomes. However despite all the interest and recent attention to the use of simulation in anesthesiology, very few studies have been able to link simulation training to improved patient outcomes [110]. Zendejas and colleagues analyzed more than 50 studies in a systemic review but they found that simulation-based education was only associated with small to moderate, nonstatistically significant patient benefits compared to nonsimulation instruction [111]. More Recently, Lorello et al. [112] carried out a meta-analysis and systemic review of 77 anesthesiology simulation studies (6066 participants). They compared simulation with no intervention (52 studies) and nonsimulation instruction (11 studies). They found that simulation in anesthesiology was more effective than no intervention (except for patient outcomes) and noninferior to nonsimulation instruction.

Even though the cost of maintaining an anesthesiology simulation lab has significantly reduced through the years, it is still a considerable burden on a very cost-conscious system. In addition to the cost there is also the need for training faculty and auxiliary staff. A recent study surveyed the radiology residency program directors to determine the factors influencing the use of high fidelity simulation at a training program. The most common reasons cited for not utilizing a high fidelity simulation in radiology residency training programs were* insufficient availability (41%) and cost (33%)* [113].

As of 2010 the American Board of Anesthesiology requires at least one simulated clinical experience per year, although most residency programs in United States have a number much higher than this [114]. Likewise one stimulated experience is required every ten years for maintenance for certification examination in anesthesiology (MOCA). The MOCA simulation course focuses not only on the medical and technical management of challenging clinical events but also on nontechnical skills of dynamic decision making and team management [115]. A review of 583 participants from first 2 years of MOCA simulation revealed that all participants (*100%*) agreed that this was* a positive learning* experience while as many as* 94%* of the participants agreed/strongly agreed that* this MOCA simulation learning experience will change their practice* [116].

The cost of implementing simulation training in anesthesiology must be justified by demonstrable improvement in patients' outcomes. Even so, the use of simulation in anesthesiology continues to grow as evident by literature; there have been more publications on this topic in the past decade than in the entire century before it. There is little doubt that the use of simulation in education will continue to grow in future. David M. Gaba, the authority on anesthesiology simulation, has summarized this notion impeccably: “No industry in which human lives depend on the skilled performance of responsible operators has waited for the unequivocal proof of the benefit of simulation before embracing it” [117].

## 13. Future of Simulation in Anesthesiology

Even though the use of simulation in anesthesiology is still a relatively new and novel development, most of the anesthesiology residency programs in US have some kind of simulation training model available. The question is not* if* the simulators will continue to be used in training of future anesthesiologist but* how* the simulators will be used. Future research should be directed to optimize the use of simulation in anesthesiology residency. This can be done by fine-tuning the simulation process by answering questions such as how often should simulation scenario be practiced, what kind of simulation devices should be used to achieve a particular learning outcomes, and what is the best possible method of debriefing after a simulation [4]. The use of simulation in an anesthesiology department requires considerable faculty development, yet such programs are poorly defined. Future research should identify the best way to approach this issue while giving due consideration to curriculum integration, clearly defined learning outcomes, and reliance on feedback [118]. Identification of the limitations of using simulation-based training and identifying situations where it would be better to resort to traditional didactic methods still remains to be defined. Over the last few years there has been an increased interest in team based simulation training particularly interdisciplinary simulation training. However, there is no definite evidence showing the benefits.

Efforts should also be directed at translating the current and future research into clinical practice. Future research should be directed at establishing a definite relationship between simulation training in anesthesiology and improved patient outcomes. In order to prove improved patient outcomes, long term, randomized, interventional studies are needed. This is necessary if residency programs and institutions are to secure financial support for the rather costly simulation infrastructure in a cost-conscious healthcare system. In summary, the use of simulation in anesthesiology is evolving rapidly and integrating deeply into the anesthesia curricula, and it seems likely it will continue to do so over the coming years.

## Figures and Tables

**Table 1:** Important milestones in simulation in anesthesiology.

Year	Simulation model	Type of model	Principle investigator/company
1960	Rescue Anne	Mechanical/physical	*Asmund Laerdal*

1965	Sim One [119]	Mechanical model with hybrid digital and analogue computer	*Dr. Stephen Abrahamson/Dr. Judson Denson* (University of Southern California)

1968	Harvey cardiology mannequin	Moderate to high fidelity model with electrical components	*Dr. Michael Gordon*

1987	Anesthesia Simulator Consultant® [30, 31]^1^	Software	*Dr. Howard A. Schwid* (Department of Anesthesiology, University of Washington)

1982	Gasman® [29, 120, 121]	Software	*Philip JH.*

1987	CASE [122]	High fidelity physical and digital model	*Dr. David Gaba*

1988	Gainesville Anesthesia Simulator [33]	High fidelity physical and digital model	*Dr. J. S. Gravenstein*

1990s	SimMan®	High fidelity physical and digital model	*Laerdal Medical*

1990s	HAL Patient Simulator	High fidelity physical and digital model	*Gaumard*® *Scientific Company*

1996	METI-Human Patient Simulator	High fidelity physical and digital model	*Medical Education Technologies Inc.*

^1^ http://anesoft.com/.
